The article "Midterm results of mitral valve repair for atrial functional mitral regurgitation: a retrospective study" was published in 2020. Journal: J Cardiothorac Surg.

# Midterm results of mitral valve repair for atrial functional mitral regurgitation: a retrospective study

**DOI:** 10.1186/s13019-020-01362-1

**Published:** 2020-10-12

**Authors:** Daisuke Kaneyuki, Hiroyuki Nakajima, Toshihisa Asakura, Akihiro Yoshitake, Chiho Tokunaga, Masato Tochii, Jun Hayashi, Akitoshi Takazawa, Hiroaki Izumida, Atsushi Iguchi

**Affiliations:** Division of Cardiovascular Surgery, Saitama Medical University International Medical Center, 1397-1, Yamane, Hidaka-shi, Saitama, 3501298 Japan

**Keywords:** Atrial functional mitral regurgitation, Atrial fibrillation, Mitral valve repair, Tricuspid ring annuloplasty, Maze procedure

## Abstract

**Background:**

Annular dilation by left atrial remodeling is considered the main cause of atrial function mitral regurgitation. Although acceptable outcomes have been obtained using mitral ring annuloplasty alone for atrial functional mitral regurgitation, data assessing outcomes of this procedure are limited. Therefore, we aimed to assess midterm outcomes of mitral valve repair in patients with atrial functional mitral regurgitation.

**Methods:**

We retrospectively studied 40 patients (mean age: 69 ± 9 years) who had atrial fibrillation that persisted for > 1 year, preserved left ventricular ejection fraction of > 40%, and mitral valve repair for atrial functional mitral regurgitation. The mean clinical follow-up duration was 42 ± 24 months.

**Results:**

Mitral ring annuloplasty was performed for all patients. Additional repair including anterior mitral leaflet neochordoplasty was performed for 22 patients. Concomitant procedures included maze procedure in 20 patients and tricuspid ring annuloplasty in 31 patients. Follow-up echocardiography showed significant decreases in left atrial dimensions and left ventricular end-diastolic dimensions. Recurrent mitral regurgitation due to ring detachment or leaflet tethering was observed in five patients and was seen more frequently among those with preoperative left ventricular dilatation. Three patients without tricuspid ring annuloplasty or sinus rhythm recovery by maze procedure developed significant tricuspid regurgitation. Five patients who underwent the maze procedure showed sinus rhythm recovery. Rates of freedom from re-admission for heart failure at 1 and 5 years after surgery were 95 and 86%, respectively.

**Conclusions:**

Mitral valve repair is not sufficient to prevent recurrent atrial functional mitral regurgitation in patients with preoperative left ventricular dilatation. Tricuspid ring annuloplasty may be required for long-term prevention of significant tricuspid regurgitation.

## Background

Left atrial (LA) dilatation and corresponding mitral annular dilatation due to long-standing atrial fibrillation (AF) may cause mitral regurgitation (MR) without left ventricular (LV) dilatation and dysfunction. This secondary functional MR has been recognized as atrial functional MR [1–5]. As annular dilation by LA remodeling has been considered the main cause of atrial function MR, mitral ring annuloplasty has been the main target of surgical intervention. However, the number of studies reporting outcomes of surgical treatment for atrial functional MR is limited [6–10]. Thus, we aimed to review the midterm outcomes of mitral valve (MV) repair for atrial functional MR.

## Methods

### Baseline characteristics

We retrospectively studied 40 patients who underwent MV repair for atrial functional MR between January 2011 and December 2018 at the Saitama Medical University International Medical Center (mean age, 69 ± 9 years; 68% male (*n* = 27)). All patients had long-standing AF that had persisted for more than 1 year, preserved LV ejection fraction (> 40%), and moderate to severe functional MR. Patients with organic valvular heart disease, including rheumatic or degenerative MV disease, a history of coronary artery disease, LV wall motion abnormality, or a history of prior cardiac surgery were excluded from the study because these conditions may confound the results. The patients’ preoperative characteristics are shown in Table 1.

**Table 1:** Preoperative patient characteristics (*n* = 40)

Covariate	Mean ± SD or Number (%)
Demographics	
Age, years	69 ± 9
Male sex	27 (68)
New York Heart Association class III/IV	3 (8)
Comorbidities	
Systemic hypertension	23 (58)
Diabetes mellitus	6 (15)
Chronic obstructive pulmonary disease	3 (8)
Chronic kidney disease	15 (38)
Cerebrovascular events	2 (5)

*SD* Standard deviation

### Echocardiography

The LA dimension, LV end-diastolic dimension, LV end-systolic dimension, and LV ejection fraction were measured [11]. The MR grade was evaluated using a multiparametric approach, including assessment of the Doppler-derived jet, effective regurgitant orifice area, MR volume and fraction, and pulmonary vein flow velocity pattern [12, 13]. The tricuspid regurgitation (TR) grade was also defined using a multiparametric approach [12, 13]. Pseudoprolapse of the anterior mitral leaflet (AML) was defined when there was a gap between the AML and the posterior mitral leaflet (PML) due to atriogenic PML tethering [8, 10, 14, 15]

### Surgical technique

Through median sternotomy, cardiopulmonary bypass was established using ascending aortic and bicaval cannulation. After sizing the intercommissural distance and AML area, an annuloplasty ring or band [semirigid Future annuloplasty band (*n* = 1), Medtronic, Minneapolis, MN; Carpentier-Edwards Physio Ring II, Edwards Lifesciences, Irvine, CA (*n* = 34); Cosgrove annuloplasty band (*n* = 3), Edwards Lifesciences; or Profile 3D (*n* = 2), Medtronic] was implanted with interrupted 2–0 Ethibond sutures. In the first half of this study, undersized ring annuloplasty was performed to address annular dilatation and increase the coaptation length. Once we understood the mechanisms of atrial functional MR, we performed true-sized ring annuloplasty to prevent aggravation of PML tethering. In the latter half of the present study, we used only a semi-rigid ring (Carpentier-Edwards Physio Ring II) larger than 28 mm. If AML pseudoprolapse existed, AML neochordoplasty was added. A pair of artificial neochordae with 4–0 or 5–0 polytetrafluoroethylene sutures (Gore-Tex sutures, W.L. Gore & Associates, Newark, DE) was placed at A2 from the anterolateral and posteromedial papillary muscle. Then, the length of the neochordae was adjusted after mitral ring annuloplasty until residual MR was diminished on water saline test. Concomitant tricuspid annuloplasty was performed in patients with severe TR, or mild or moderate TR with a dilated annulus (≥40 mm or > 21 mm/m^2^ by transthoracic echocardiography) [16]. A tricuspid annuloplasty ring [MC3 ring (*n* = 17), Edwards Lifesciences; Physio Tricuspid annuloplasty ring (*n* = 10), Edwards Lifesciences; Contour 3D annuloplasty ring (*n* = 3), Medtronic; or a Tri-Ad Adams tricuspid annuloplasty ring (*n* = 1), Medtronic] was implanted with interrupted 2–0 Ethibond sutures. The indication of the maze procedure and LA plication was decided at surgeon’s discretion based on the period of atrial fibrillation and the size of LA.

### Follow-up

Clinical follow-up examinations were completed for all patients. The mean follow-up period was 42 ± 24 months. Follow-up echocardiography was performed 1 week after surgery and every year after discharge. The mean echocardiographic follow-up period was 26 ± 24 months.

### Statistical analyses

Descriptive statistics were reported as the mean ± standard deviation for continuous variables and as frequencies and percentages for categorical variables unless otherwise noted. A comparison between the groups was performed using Student’s *t* test or Wilcoxon-Mann-Whitney *U*-test for continuous variables and the chi-square or Fisher’s exact test for categorical variables. Event-free rates were estimated using Kaplan-Meier analysis. *P*-values < 0.05 were considered to indicate statistical significance. Statistical analyses were performed using JMP software (version 14.1.0; SAS institute, Cary, NC).

## Results

### Echocardiographic outcomes

The mean LV end-systolic dimension and mean LV ejection fraction did not significantly change between the preoperative period and the follow-up period. The mean LA dimension significantly decreased from the preoperative period (60 ± 11 mm) to the follow-up period (54 ± 13 mm, *p* < 0.001). The mean LV end-diastolic dimension significantly decreased from the preoperative period (55 ± 7 mm) to the follow-up period (51 ± 8 mm, *p* < 0.001).

All patients were discharged with an MR grade no greater than mild, except one patient with moderate MR. During the follow-up period, four patients developed moderate or severe MR. Two patients with end-stage renal disease who underwent mitral ring annuloplasty alone with a 26-mm Cosgrove annuloplasty band and a 28-mm Physio Ring II developed severe MR due to partial detachment of prosthetic rings. Other patients developed moderate or severe MR due to PML tethering (Table 2). One of these patients underwent mitral ring annuloplasty with PML augmentation and basal chordae resection. Two other patients underwent mitral ring annuloplasty with AML neochordoplasty on initial surgery.

**Table 2:** Preoperative and follow-up echocardiographic data (*n* = 40)

	Preoperative data	Follow-up data	***P*** value
LA dimension (mm)	60 ± 11	54 ± 13	<.001*
LV end-diastolic dimension (mm)	55 ± 7	51 ± 8	<.001*
LV end-systolic dimension (mm)	37 ± 7	36 ± 9	0.30
Ejection fraction (%)	60 ± 11	57 ± 15	0.13
Moderate or severe MR	40	5	
Moderate or severe TR	22	3	

*LA* Left atrial, *LV* Left ventricular, *MR* Mitral regurgitation, *TR* Tricuspid regurgitation

*statistically significant

Table 3 shows the preoperative transthoracic echocardiography data of patients who developed recurrent MR (*n* = 5) and those without MR recurrence (*n* = 35). Mean LA dimensions, mean LV end-diastolic dimensions, and mean LV end-systolic dimensions were significantly larger in patients with recurrent MR than in patients without recurrent MR.

**Table 3:** Preoperative echocardiographic data for patients with and without recurrent MR (*n* = 40)

	Recurrent MR (+)	Recurrent MR (−)	***P*** value
LA dimension (mm)	71 ± 12	59 ± 9	0.008*
LV end-diastolic dimension (mm)	64 ± 3	54 ± 1	0.001*
LV end-systolic dimension (mm)	43 ± 3	36 ± 1	0.034*
Ejection fraction (%)	60 ± 5	60 ± 2	0.91

*LAD* Left atrial, *LV* Left ventricular, *MR* Mitral regurgitation

*statistically significant

Receiver-operating characteristic curves were used to evaluate the cutoff values of LV end-diastolic dimensions as a preoperative predictor for recurrent moderate or severe MR. LV end-diastolic dimensions of 61 mm had a sensitivity of 91% and a specificity of 80% for predicting recurrent moderate or severe MR. The area under the curve for LV end-diastolic dimensions was 0.897 (Fig. 1).

**Fig. 1:** Receiver operating characteristic curve showing LV end-diastolic dimension as a predictor of recurrent moderate or severe mitral regurgitation in patient with atrial functional mitral regurgitation. The LVDd of 61 mm had a sensitivity of 91% and a specificity of 80% for predicting recurrent moderate or severe mitral regurgitation. The area under the curve for LV end-diastolic dimension was 0.897. LV = left ventricular

Moderate or severe TR was found in 22 patients preoperatively. All patients were discharged with a TR grade no greater than mild. However, among five patients without tricuspid ring annuloplasty or sinus recovery by maze procedure, three patients developed moderate or severe recurrent TR during the follow-up period.

### Perioperative data

All patients underwent mitral ring annuloplasty. The median size of the implanted ring was 28 mm (range: 24–32 mm). As determined by intraoperative observation, mechanisms of MR included annular dilatation alone in 19 patients and annular dilatation with AML pseudoprolapse in 19 patients. Additional MV repair was performed for 22 patients, which included AML neochordoplasty in 19 patients, PML augmentation in 3, and basal chordae resection in 2. Other concomitant procedures included the maze procedure in 20 patients, tricuspid ring annuloplasty in 31, and LA plication in 9. These data are summarized in Table 4.

**Table 4:** Operative patient characteristics (*n* = 40)

Covariate	Mean ± SD or Number (%)
Median annuloplasty ring size (range)	28 (24–34) mm
Mitral valve procedures	
Mitral ring annuloplasty only	19 (48)
Anterior mitral leaflet neochordoplasty	19 (48)
Posterior mitral leaflet augmentation	3 (8)
Basal chordae resection	2 (5)
Concomitant procedures	
Maze procedures	20 (50)
Tricuspid ring annuloplasty	31 (78)
Left atrial plication	9 (23)
Cardiopulmonary bypass time	177 ± 38 min
Cross-clamp time	134 ± 31 min

*SD* Standard deviation

### Clinical outcomes

There were no cases of in-hospital mortality. Postoperative complication included acute renal failure requiring hemodialysis in two patients, re-exploration for bleeding in one patient, and stroke in one patient. Among the 20 patients who underwent the maze procedure, sinus rhythm was recovered in five patients (25%).

During the follow-up period, one patient experienced stroke due to infective endocarditis resulting in heart failure, seven patients required re-admission because of worsening heart failure, and six patients required permanent pacemaker implantation for sick sinus syndrome. Among five patients with recurrent MR, two patients with ring detachment required reoperation for prosthetic valve replacement 37 months and 63 months after initial operations. Seven patients died during the follow-up period because of congestive heart failure (four patients) and pneumonia (three patients) (Table 5). The rates of freedom from recurrent MR were 97.1% at 1 year, 85.4% at 3 years, and 62.3% at 5 years after surgery (Fig. 2). The rates of freedom from re-admission for heart failure were 94.9% at 1 year, 85.7% at 3 years, and 85.7% at 5 years after surgery (Fig. 3).

**Table 5:** Early and midterm clinical outcomes (*n* = 40)

Covariate	Mean ± SD or Number (%)
Early outcomes	
In-hospital mortality	0
Acute renal failure requiring hemodialysis	2 (5)
Re-exploration for bleeding	1 (3)
Cerebrovascular events	1 (3)
Deep sternal wound infection	0
Midterm outcomes	
Patient deaths during the follow-up period	7 (18)
Cardiac death	4 (10)
Recurrent moderate or severe MR	5 (13)
Re-admission for heart failure	7 (18)
Cerebrovascular events	1 (3)
Reoperation for recurrent MR	2 (5)
Permanent pacemaker implantation	6 (15)
Systemic embolism	1 (3)

*MR* Mitral regurgitation, *SD* Standard deviation

**Fig. 2:** Freedom from recurrent moderate or severe mitral regurgitation (MR)

**Fig. 3:** Freedom from re-admission for heart failure

## Discussion

This study investigated midterm outcomes after MV repair for atrial functional MR. Although atrial functional MR was shown to have been repaired successfully on postoperative echocardiography, some patients with preoperative LV dilatation developed recurrent MR due to prosthetic ring detachment or PML tethering during the follow-up period resulting in heart failure and cardiac death. In addition, only 25% (5/20) of the patients who underwent maze procedures showed sinus rhythm recovery, and 60% (3/5) of the patients without sinus rhythm recovery or tricuspid ring annuloplasty developed moderate or severe TR.

Atrial functional MR can be mitigated using sinus rhythm restoration strategies via reverse LA anatomical and mechanical remodeling [17]. Some patients, especially with a giant LA and long-standing AF may be refractory to catheter ablation. As the LA volume continues to increase with persistent AF, patients can develop congestive heart failure that cannot be managed with medications. Although surgical indication for atrial functional MR remains uncertain, surgical intervention has been reported to be beneficial for decreasing LA volume, severity of MR, and clinical symptoms in heart failure [6–10]. In addition, this study showed decreased LA dimension and LV end-diastolic dimension on follow-up echocardiography.

The main surgical strategy for atrial functional MR was to repair mitral annular dilatation with ring annuloplasty. Five patients developed recurrent MR during the postoperative and follow-up periods. One cause of recurrent MR was prosthetic ring detachment, which was common in patients with end-stage renal disease. Because expansion of the LA wall leads to deviation of the posterior annulus toward the outside of the myocardium [18, 19], placing the sutures correctly within the posterior annulus may be challenging. Further, LA and mitral annular dilatation worsened if AF was sustained in this study. This may increase the tension between the prosthetic ring and the posterior mitral annulus. Another cause of recurrent MR was PML tethering. Although AML neochordoplasty, PML augmentation, and basal chordal resection was performed to repair AML pseudoprolapse or atriogenic PML tethering, recurrent MR due to PML tethering was not completely prevented. This study revealed that preoperative echocardiography in patients with recurrent MR showed LV dilatation. This finding was in line with that of a previous study [9]. LV dilatation is a morphological change in the late phase of atrial functional MR. Therefore, surgical intervention before the late phase may be beneficial. Otherwise further additional repair including subvalvular apparatus procedures or mitral valve replacement may be required in patients in the late phase of atrial functional MR.

Long-standing AF is also known to cause functional secondary TR due to tricuspid annular dilatation [20]. Takahashi et al. suggested that MV repair in addition to tricuspid valve repair should be considered because atrial functional MR and TR are dual-valve diseases [10]. The present study showed that 60% of the patients without tricuspid ring annuloplasty or sinus rhythm recovery using the maze procedure developed moderate or severe TR during the follow-up period. Because the efficacy of the maze procedure in patients with significant LA dilatation was limited [21], tricuspid ring annuloplasty should be performed in addition to MV repair for atrial functional MR.

The indication of the maze procedure for patients with atrial functional MR remains unclear. Patients with a giant LA and long-standing AF who are refractory to catheter ablation are also usually refractory to the maze procedure. However, restoration of sinus rhythm is the fundamental treatment for atrial functional MR and some patients can receive benefits from the maze procedure. The balance of benefits and risks of the maze procedure should be taken into consideration, and further study should elucidate the reasonable indication of the maze procedure. Although the indication of LA plication also remains unclear, Takahashi et al. [10] reported that one patient showed a gradual increase in the LA volume index, and this resulted in re-worsening of the PML tethering. Therefore, LA plication might prevent further PML tethering. In addition, Wang et al. [22] showed that overall restoration of sinus rhythm was significantly improved in the group with aggressive reduction of LA wall tension during a 1-year clinical follow-up. They concluded that aggressive LA size reduction might be a key factor for maintenance of sinus rhythm after the maze procedure. Because sinus rhythm recovery is one of key factors to prevent atrial functional MR progression, LA plication may be beneficial.

### Limitations

This study has several limitations. This was a single-center, retrospective observational study with a small number of patients. The use of multiple mitral annuloplasty rings was a major confounding variable. All control subjects underwent additional MV repair for AML pseudoprolapse or PML tethering. Thus, studies with longer follow-up periods and more statistical power are essential to validate the performance of additional MV repair for atrial functional MR. Moreover, echocardiographic studies using transesophageal echocardiography with three-dimensional morphological analysis are warranted to acquire more accurate data and to elucidate further mechanisms of recurrent MR. Finally, this study included patients with preoperative LV dilatation, which may be associated with ventriculogenic tethering. Although some argue that atriogenic and ventriculogenic should be differentiated, there is still no clear definition of atrial functional MR, and we believe that LV dilatation is one mechanism underlying the severe form of atrial functional MR. Therefore, studying the entire spectrum of atrial functional MR is crucial to elucidate the optimal surgical timing and technique.

## Conclusions

Our analysis suggests that recurrent MR due to prosthetic ring detachment or PML tethering occurred even after mitral ring annuloplasty with additional repair techniques in patients with atrial functional MR and preoperative LV dilatation. Because sinus rhythm recovery was not sufficient after the maze procedure in patients with severe LA dilatation, tricuspid ring annuloplasty is recommended for patients without considerable operative risk.

## Data Availability

The datasets used and analyzed during the current study are available from the corresponding author on reasonable request.

## Abbreviations

AF: Atrial fibrillation
AML: Anterior mitral leaflet
LA: Left atrium
LV: Left ventricle
MR: Mitral regurgitation
MV: Mitral valve
PML: Posterior mitral leaflet
TR: Tricuspid regurgitation
